# mTORC2 regulates hedgehog pathway activity by promoting stability to Gli2 protein and its nuclear translocation

**DOI:** 10.1038/cddis.2017.296

**Published:** 2017-07-13

**Authors:** Samarpan Maiti, Susmita Mondal, Eswara M Satyavarapu, Chitra Mandal

**Affiliations:** 1 Cancer Biology and Inflammatory Disorder Division, Council of Scientific and Industrial Research (CSIR)-Indian Institute of Chemical Biology, 4, Raja S.C. Mullick Road, Jadavpur, Kolkata 700032, India

## Abstract

mTORC2 is aberrantly activated in cancer and therefore is considered to be an important therapeutic target. The hedgehog pathway, which is also often hyperactivated, regulates transcription of several genes associated with angiogenesis, metastasis, cellular proliferation and cancer stem cell (CSC) regeneration. However, the contribution of mTORC2 toward hedgehog pathway activity has not been explored yet. Here we have addressed the molecular cross talk between mTORC2 and hedgehog pathway activities in the context of glioblastoma multiforme, a malignant brain tumor using as a model system. We observed that higher mTORC2 activity enhanced the expression of a few hedgehog pathway molecules (Gli1, Gli2 and Ptch1) and amplified its target genes (Cyclin D1, Cyclin D2, Cyclin E, Snail, Slug and VEGF) both in mRNA and protein levels as corroborated by increased metastasis, angiogenesis, cellular proliferation and stem cell regeneration. Inhibition of mTORC2 formation decreased hedgehog pathway activity and attenuated all these above-mentioned events, suggesting their cross talk with each other. Further investigations revealed that mTORC2 inhibited ubiquitination of Gli2 by inactivating GSK3*β*, and thus it promotes stability to Gli2 and its nuclear translocation. Moreover, enhanced mTORC2 activity led to the increased clonogenic properties and CD133^+^ cells, indicating its role in CSC regeneration. mTORC2 inhibitor directed the reduction of hedgehog pathway proteins and also reduced CSCs. Thus, our observations support a role for elevated mTORC2 activity in regulating angiogenesis, metastasis, cellular proliferation and CSC regeneration via hedgehog pathway activity. Taken together, it provides a rationale for including the mTOR2 inhibitor as part of the therapeutic regimen for CSCs.

Glioblastoma multiforme (GBM) represents the most common form of malignant brain tumors in adults with extremely low survival rate.^1^ Deregulation of mTORC2 signaling is one of the main mechanisms in GBM formation.^2^ Hyperactivation of mTORC2 with Rictor overexpression was found to cause GBM.^3, 4^ mTORC2 has been linked with several metabolic reprogramming activities and is a major regulatory molecule.^5, 6^

The hedgehog (Hh) pathway is another major regulator of cellular differentiation, proliferation and stem cell maintenance. Aberrant activation of the Hh pathway is associated with GBM and leads to the activation of cancer stem-like cells (CSCs).^7^ Transcriptional activation of Hh target genes occurs through the actions of Gli1, Gli2 and Gli3 (ref. 8). Gli1 acts as a transcriptional activator and is also regulated by Gli2 (ref. 9), whereas Gli2 and Gli3 act as both transcriptional activators and repressors based on post-translational modification. Evidence suggests that the full-length form of Gli2 proteins (Gli2^FL^) acts as a strong activator of Hh signaling.^10^ Upon stabilization, Gli2 moves in the nucleus, which in turn promotes the transcription of both Gli1 and Gli2 and amplifies the transcription of other target genes.

CSCs are considered the origin of tumorigenesis, drug resistance and relapse recurrence.^11, 12^ They display persistent activation of one or more highly conserved hedgehog, Notch and Wnt signal transduction pathways. Therefore, CSCs are important targets for therapeutic intervention.

Keeping in view the aberrant activation of both Hh and mTORC2 pathways and their role in GBM formation, there are needs to explore their contextual functioning in depth (Figure 1a). It will be useful to distinguish some specific molecules that are common to these pathways that can serve as potential drug targets. Here we have demonstrated a positive correlation between mTORC2 activity and Hh-pathway upregulation, leading to more invasiveness, angiogenesis and cellular proliferation of GBM cells. Furthermore, we have observed that the interaction between mTORC2 and Hh-pathway molecules is associated with increased stemness properties. More importantly, we showed that inhibitors that target mTORC2 also target the Hh pathway and reduce the cell viabilities of CSCs.

## Results

### Differential mTORC2 activity leads to disparity in expression of Hh pathway proteins in GBM cells

To understand the impact of mTORC2 activity in the regulation of the Hh pathway, we selected two GBM cell lines namely U87MG and LN229 (Figure 1a). Previously, we reported that mTORC2 activity is higher in the U87MG compared with the LN229 (Supplementary Figure S1).^13^ Here, we observed the enhanced level of Gli1, Gli2^FL^ and Ptch1 proteins in U87MG compared with LN229 (Figure 1b). Gli3 repressor (Gli3^Rep^) expression was lower in U87MG. However, no apparent changes of other Hh-pathway proteins Sufu, Smo and Shh were observed.

These changes in protein level of Gli1, Gli2^FL^, Gli3^Rep^ and Ptch1 made us curious to know what was happening in genetic expression. We checked the mRNA level and observed the lower genetic expression of all four molecules in LN229 compared with U87MG (Figure 1c). This observation led us to think that some relationship possibly exists between mTORC2 activity and Hh-pathway proteins.

To understand this relationship, we used Rictor_1 and Rictor_2 shRNAs that suppress the expression of Rictor to block the activity of mTORC2 in U87MG cells. Coimmunoprecipitation and western blot analysis showed lower mTORC2 formation and reduced mTOR Ser2481 phosphorylation, a signature of active mTORC2 as we showed earlier (Figure 2a).^13^ In such a condition, we found that there were reduced expressions of Gli1, Gli2 and Ptch1 at the genetic level (Figure 2b), as well as at the protein level (Figure 2c). However, Gli3 was also reduced at the gene level, but its repressor forms increased at the protein level.

In addition, mTORC2 formation was also promoted in LN229 cells by overexpressing Rictor with myc-tag wild-type Rictor (pRK-5/Rictor) as we did earlier.^13^ We found enhanced mTOR Ser2481 phosphorylation and higher association of mTOR and Rictor by coimmunoprecipitation (Figure 2d). This enhanced mTORC2 activity in Rictor-overexpressed cells led to the increase of Gli1, Gli2, Gli3 and Ptch1 at the genetic level (Figure 2e) and also at the protein level (Figure 2f). Such observations strengthened our hypothesis that mTORC2 and Hh pathway are interconnected.

For further confirmation, we transfected both U87MG and LN229 with Gli reporter construct and checked its expression by luciferase assay (Figure 2g). We observed higher expression of Gli reporter genes in U87MG compared with LN229, suggesting a connection of the Hh pathway with the differential basal level of mTORC2 activity. Furthermore, Rictor was either knocked down or overexpressed in Gli reporter-transfected U87MG or LN229, respectively. Results showed that expression of Gli reporter genes was decreased when Rictor was knocked down in U87MG. In contrast, Rictor-overexpressed LN229 exhibited increased expression of Gli reporter gene. In addition, this enhanced expression of Gli reporter gene was reduced in the presence of Hh inhibitor Gant 61. Taken together, our observation strongly supports the role of mTORC2 activity in regulation of the Hh pathway.

### mTORC2 regulates cellular proliferation, angiogenesis, invasion and metastasis through the Hh pathway

To confirm the upstream regulation of Gli1 and Gli2 by mTORC2, we examined the expression of a few important target genes of these two molecules by reducing the mTORC2 activity in U87MG or enhancing the mTORC2 activity in LN229. Slug and snail are known to be responsible for invasion and migration, whereas VEGF helps in angiogenesis. Rictor-knocked-down U87MG exhibited reduced Slug, Snail and VEGF both at genetic (Figure 3a) and protein levels (Figure 3c). Similarly, the levels of all three molecules were enhanced in Rictor-overexpressed LN229 (Figures 3b and c). These observations were further corroborated by *in vitro* invasion, migration and angiogenesis profiles in U87MG and LN229 under different conditions (Figures 3d–h).

We compared the ability of connective tube formation, which is a signature of angiogenesis. We found that within 72 h U87MG can form the thread-like connections between themselves compared with LN229 (Figure 3d). However, when Rictor was knocked down, U87MG showed no connective tube formation after 72 h. A similar situation was observed when cells were treated with Hh inhibitor. In contrast, LN229 that did not show connective tube formation ability within 72 h was able to form connective tubes upon Rictor overexpression. However, this Rictor-driven connective tube formation was inhibited in the presence of Hh inhibitor.

The invasion ability was monitored both in Rictor-knocked down and in overexpressed conditions using matrigel-coated insert systems (Figures 3e and f). Cells that invade the membrane adhered to the lower surface were stained with crystal violet. Three randomly selected fields on the lower side of the insert were photographed, and the migrated cells were counted. We found that U87MG can invade matrigel within 48 h (Figure 3e). However, when Rictor was knocked down or cells were treated with Hh inhibitor, they cannot invade the matrigel after 48 h. In contrast, LN229 cells that had poor invasion ability showed higher invasion capability when the mTORC2 formation was induced. These Rictor-overexpressed LN229 cells again showed lower invasion in the presence of Hh inhibitors (Figure 3e).

Next, we checked the cellular migration ability of these cells by scratch wound assay (Figures 3g and h). We found that U87MG can fill the gap, whereas LN229 cannot even after 36 h (Figure 3g). However, upon Rictor knockdown or treatment with Hh inhibitors, U87MG showed decreased migration ability. In contrast, LN229 showed increased migration capability upon promoting mTORC2 activity by Rictor overexpression. However, migration potential was reduced when Rictor-overexpressed LN229 was treated with Hh inhibitor.

Furthermore, we checked the status of a few cell cycle regulatory proteins whose expressions are known to be regulated by Gli1 and Gli2 proteins in the Hh pathway (Figures 3i–k). We observed that when mTORC2 activity is reduced in U87MG cells by silencing Rictor, there was diminution of cyclin D1, cyclin D2 and cyclin E at mRNA and protein levels (Figures 3i and k). Similarly, Rictor-overexpressed LN229 cell with enhanced mTORC2 activity exhibited improved levels of these cell cycle regulatory proteins (Figures 3j and k). To strengthen our findings, we checked the cell cycle status and found enhanced G0/G1 cell cycle arrest in Rictor-knocked-down U87MG cells (Figure 3l). In addition, there was an enrichment of cells in the M phase when mTORC2 activity was induced in LN229. All these data support that mTORC2 activity is required for cell cycle regulation via Gli1/Gli2.

### mTORC2 regulates the Hh pathway via GSK3*β* and promotes nuclear translocation of Gli2 proteins

So far we have established a close relationship between mTORC2 activity and upregulation of the Hh pathway. GSK3*β* is known to play an important role in regulating the Hh pathway. Previously it was reported that mTORC2 and GSK3*β* have reciprocal activation in cancer including GBM.^13^ Upon Rictor knockdown, inhibitory phosphorylation of GSK3*β* at Ser9 was increased in U87MG cells and decreased in Rictor-overexpressed LN229 cells, as we have seen earlier (Figure 4a).^13^ Here we have addressed an obvious question whether mTORC2 plays as a master molecule in regulating the Hh pathway via GSK3*β* (Figure 4b). Rictor-knocked-down U87MG cells exhibited decreased levels of Gli1, Gli2^FL^ and Ptch1, as observed in Figure 2c. However, when we silenced both Rictor and GSK3*β*, we observed enhancement of these three molecules (Figure 4b). In contrast, GSK3*β*-knocked-down LN229 cells exhibited increased levels of Gli1, Gli2^FL^ and Ptch1, suggesting that GSK3*β* is responsible for the stability of these proteins. However, after Rictor overexpression and simultaneously GSK3*β* knockdown, these cells show more increased levels of Gli2^FL^, Gli1 and Ptch1 compared with control or only GSK3*β*-knocked-down LN229 cells. Therefore, it suggests that GSK3*β* possibly plays an interconnecting molecule between mTORC2 and the Hh pathway.

When GSK3*β* is active, it phosphorylates Gli2 and phosphorylated Gli2 is then directed for ubiquitination. Accordingly, we wanted to check whether Gli2 is getting degraded via the GSK3*β*-mediated ubiquitination pathway in LN229 cells. To demonstrate that, we treated LN229 cells either with MG132 to block the protein ubiquitination or with GSK3*β* inhibitor separately (Figure 4c). We found that in both the cases there were enhancements of Gli2^FL^ level in a dose-dependent manner, suggesting that Gli2^FL^ degradation via GSK3*β* is the reason for lower Gli2^FL^ level in these cells.

To further corroborate, we overexpressed the Gli2^FL^ construct (pCS2-MT GLI2 FL) in LN229 so that the Gli2 accumulation in a cell becomes higher. We found an enhanced level of Gli2 protein, which further leads to activation of other Hh pathway molecules such as Gli1 and Ptch1, as well as downstream target molecules such as Cyclin D1, Cyclin D2, VEGF, Snail and Slug both at mRNA and protein levels (Figures 4d and e). All these observations clearly demonstrated that Gli2 degradation is one of the prime reasons for lowering the Hh pathway activity in LN229 cells.

So far we observed that the expression levels of Hh pathway molecules and its target genes were lower in LN229 compared with U87MG cells (Figure 3). This may be because of the probable hindrances in the transcription of those genes. Therefore, we checked the translocation of Gli1 and Gli2 from the cytoplasm to the nucleus. Here we observed the reduced nuclear localization of Gli2 and Gli1 in LN229 cells compared with U87MG (Figure 4f). This might be possible because of restriction imposed by some other molecules for their translocation into the nucleus.

Sufu, another important Hh pathway protein, associates with Gli1/Gli2 and prevents its nuclear accumulation through cytoplasmic retention. GSK3*β*, when active, phosphorylates sufu and the phosphorylated form of sufu binds with Gli1/Gli2 to form the Sufu–Gli1/Gli2 complex. Here we observed that in LN229 GSK3*β* is more active compared with U87MG. Accordingly, Sufu would be more stable in LN229 and will form abundant Sufu–Gli2 complex. As expected, we observed higher Sufu–Gli2 complexes compared with U87MG as revealed by the coimmunoprecipitation study (Figure 4g). These data further strengthen our observation that mTORC2 modulates the activity of Hh pathway target genes by restricting the Gli1/Gli2 translocation into the nucleus.

For further interaction between molecules of mTORC2 and the hedgehog pathway, we carried out the coimmunoprecipitation study and identified the binding of Rictor with both Sufu and Smo among all of the hedgehog pathway molecules (Figure 4h). However, it demonstrated differential association based on mTORC2 activity. Rictor exhibited higher association with Sufu in LN229, whereas Rictor-Smo binding was more in U87MG cells, suggesting that there might be some other mechanism that also modulates the Hh pathway.

### mTORC2 regulates the stemness of GBM cells via the hedgehog pathway

So far we have demonstrated mTORC2 as a key to the Hh pathway (Figures 1, 2, 3, 4); next, we wanted to address its role in the stemness of GBM cells. From U87MG cells, we isolated enriched population of stem-like cells that showed larger colony and enhanced expression of CD133, Nestin, Oct4, Sox2 and Nanog (Supplementary Figure S2).

These stem-like cells exhibited increased mTORC2 activity as indicated by higher mTOR Ser2481 phosphorylation (Figure 5a). They also showed higher association of Rictor with mTOR, indicating more mTORC2 formation compared with U87MG. Next, we cultured SVG cells (normal human glial cells) in stem cell medium and isolated the colonies that we considered as normal human stem-like cells. These cells showed lower mTOR Ser2481 phosphorylation and Gli2 protein levels compared with CSCs, suggesting a role of Gli2 and mTORC2 activity in CSC generation (Figure 5b).

To further confirm the contribution of mTORC2 in induction of stemness property, we overexpressed rictor in LN229 cells and found large numbers of neurospheres formation and increased expression of CD133, Oct4, Sox2, Nanog, Nestin and Integrin 6 (Figures 5c–e). However, these rictor-overexpressed cells were unable to form neurospheres when Gli2 was knocked down. Such observations point toward the fact that mTORC2 is responsible for the stemness properties of cancer cells through the hedgehog pathway.

### mTORC2 is a potent target to promote apoptosis of CSCs

So far we have observed that the stemness properties are maintained by mTORC2 (Figure 5). We have also demonstrated involvement of mTORC2 and hedgehog pathway in migration, invasion, angiogenesis and proliferation (Figure 3). Accordingly, we hypothesize that a good mTORC2 inhibitor would help to reduce the CSCs by targeting all these hedgehog pathway activities (Figure 6).

We then selected a few inhibitors that target either mTORC2 (KU-0063794) or Shh (cyclopamine) or Gli2 (Gant61) or a known drug for GBM (temozolomide). In addition, we have also used a newly identified carbazole alkaloid, mahanine, as an mTORC1/2 inhibitor.^13^ Next, CD133+ stem-like cells were treated with these inhibitors at different doses for 48 h. Both mahanine and KU-0063794 exhibited highest dose-dependent increase in cell mortality in comparison with others (Figure 6a). Therefore, it suggested that mTORC2 could be a better therapeutic target for GBM stem-like cells.

Therefore, we wanted to explore the molecules/events to target CSCs by an mTORC1/2 inhibitor. As mahanine showed better efficacy to reduce CSCs, we selected this molecule for further study. Mahanine-treated U87MG cells exhibited reduced Gli1 and Gli2^FL^ proteins in a dose-dependent manner, suggesting mTORC2 as a key target to hit the hedgehog pathway (Figure 6b). Furthermore, we found that mahanine-treated GBM stem-like cells were unable to form neurospheres (Figure 6c), exhibited reduced CD133^+^ cells in culture (Figure 6d) and exhibited dose-dependent cytotoxicity as determined by increased PI positivity (Figure 6e) with minimum toxicity to normal stem-like cells (Figure 6f).

## Discussion

We have investigated molecular regulation and cross talk between mTORC2 and hedgehog pathway and its therapeutic implication in the GBM model. The key achievement of our study is providing evidence that mTORC2 plays a major regulatory molecule for the activation of the hedgehog pathway. It stabilizes Gli2 by inhibiting GSK3*β*. Consequently, it promotes nuclear translocation of Gli2. This was reflected in enhanced metastasis, angiogenesis and cellular proliferation because of increased hedgehog pathway activity through mTORC2 formation. In addition, we have observed that mTORC2 activity is required for the stemness properties of GBM cells and established mTORC2 to be a better therapeutic target in CSCs. All these events have been demonstrated pictorially in Figure 6g. To the best of our knowledge, this is the first evidence demonstrating molecular cross-talk between mTORC2 and the hedgehog pathway.

Aberrant hedgehog pathway activity and mTORC2 upregulation are always associated with high-grade GBM formation.^14, 15^ TCGA-GBM database analysis suggests a strong correlation between Gli1, Gli2, Gli3 and Ptch1 mRNA expression and hedgehog pathway activity in GBM formation.^16^ In a Drosophila model, loss of functional Rictor and SIN1 alleles prevented glioma formation, demonstrating requirement of mTORC2.^17^ Cumulatively, all these correlation patterns are suggestive of the necessity of both the canonical Hh pathway and mTORC2 activities in GBM.

Our in-depth study demonstrated that in GBM cells, where mTORC2 was activated, the hedgehog pathway also activated as evidenced by upregulation of Gli1, Gli2^FL^, Ptch1 and the downstream target genes (VEGF, Slug, Snail, Cyclin D1, Cyclin D2, Cyclin E). It was further supported by the observation that disruption of mTORC2 formation decreased the levels of all these proteins. Gli2 is known to be responsible for the transcriptional expression of Gli2 itself and both Gli1 and Ptch1.^18^ Gli2 and Gli1 both are then accountable for transcription of Slug, Snail, VEGF, Cyclin D1, Cyclin D2, Cyclin E and many others^19^ whereas full-length Gli3 (molecular weight 190 kD) acts as an activator of transcription while in the absence of Hh signaling it is cleaved to form a truncated repressor (molecular weight 83 kDa).^18^ However, in our system, we found that upon mTORC2 disruption Gli3 expression decreased at the gene level but its repressor form Gli3^Rep^ was increased. This also indicated that mTORC2 disruption inhibited Hh signaling.

For further confirmation, we have assessed quantitatively the activity of Gli reporter genes in a different cellular perspective. Where mTORC2 was less active the expression of Gli Reporter activity was also low, and the expression was increased when Rictor was overexpressed. Moreover, when Gli2 activity was blocked, mTORC2-dependent Hh-pathway activity decreased in spite of Rictor overexpression. This strongly supports that mTORC2 regulates transcription of Gli2 target genes.

Proteolytic processing of Gli2 protein is extremely inefficient. Therefore, the majority of Gli2 protein exists as a full-length form.^20^ Small fraction of processed Gli2 also rapidly degraded, which is mainly dependent on the phosphorylation of four PKA and multiple adjacent CK1 and GSK3 sites.^20, 21^ GSK3/CK1 phosphorylation sites are required for the proteolysis of Gli2. The hyperphosphorylation of Gli2 protein triggers ubiquitination and proteasome-mediated protein degradation.^22^

mTORC2 is known to inactivate GSK3*β*,^13^ and as a consequence it cannot phosphorylate Gli2 for ubiquitination, expecting more accumulation. Interestingly, we observed enhanced Gli2^FL^, Gli1 and Ptch1 even in Rictor-knocked-down U87MG and also in Rictor-overexpressed LN229 cells when GSK3*β* were silenced. Reports indicated that mutant Gli2 lacking GSK3 and CK1 sites is hyperactive.^22^ Therefore, it may be envisaged that GSK3*β* plays as an interconnecting molecule between mTORC2 and Hh pathway.

Involvement of GSK3*β* was further proved when we found that GSK3*β* inhibitor led to the accumulation of Gli2^FL^ in cells. Blocking of proteosome also rescued Gli2^FL^ accumulation. This helped us to conclude that mTORC2 inhibits proteasomal degradation of Gli2^FL^ via GSK3*β* inactivation. When Gli2^FL^ is stable, it translocates into the nucleus and promotes the transcription of Gli1/Gli2^FL^ and other target genes.

Sufu is an essential negative regulator of the Hh pathway.^23, 24^ It is phosphorylated at Ser-342 and Ser-346 by GSK3*β*.^25^ Phosphorylated Sufu forms stable Sufu–Gli complex, and thereby nuclear translocation of Gli proteins is restricted. Dephosphorylated Sufu is degraded by the ubiquitin–proteasome system. Our observation confirmed higher GSK3*β* activity in LN229. As expected, we also found that Sufu is highly associated with Gli2^FL^ which was reflected with the lower genetic expression of Gli1, Gli2^FL^ and Ptch1.

We also found that Rictor itself interacted directly with Smo and Sufu. However, the association between Rictor and Sufu was higher where mTORC2 formation was lower. Previously, we observed almost an equivalent amount of Rictor both in U87MG and LN229.^13^ Therefore, it might be possible that as in LN229 mTORC2 formations are lower there may be free Rictor that was available for binding with Sufu and giving stability to the Sufu–Gli2 complex. We also found that Rictor exhibited higher binding with Smo in U87MG compared with LN229, which possibly reflected in the higher activation of the Hh pathway in U87MG irrespective of a conventional Shh ligand. However, it needs more in-depth studies to understand such differential binding.

Hh pathway and mTORC2 are both known to be involved in invasiveness, metastasis and angiogenesis.^26, 27, 28^ Our findings support that mTORC2-mediated metastasis, invasion and angiogenesis actually happened by the activation of the Hh pathway, which in turn promotes the genetic expression of Snail, Slug and VEGF. In contrast, when the Hh pathway was inhibited, mTORC2 activity alone was unable to promote these events.

Xenograft studies using rictor-overexpressing/rictor-knockdown cells supported a role for increased mTORC2 and cell cycle activities.^3^ Ectopic expression of Gli2 in nontumorigenic prostate epithelial cells resulted in accelerated cell cycle progression.^29^ Here we showed that mTORC2-mediated increased Hh pathway activity promotes transcription of several cell cycle regulatory proteins (Cyclin D1, Cyclin D2 and Cyclin E), which is responsible for increased proliferation.

Our observation of contextual functioning of mTORC2 and the Hh pathway also suggests that mTORC2 might have a role in the regulation of CSCs through the Hh pathway. Indeed, mTORC2 formation and activity were higher in CSCs compared with non-stem cancer cells. Cells that are unable to form CSC colonies are able to generate a significantly higher number of large colonies when transfected with exogenous Rictor. These Rictor-transfected cells also showed higher stemness property. However, all these stemness characteristics were hindered in Rictor-transfected cells when Hh signaling was inhibited, suggesting regulation of stemness in GBM by mTORC2 via the Hh pathway.

In addition, we observed higher mTORC2 activity in the GBM-stem-like cell compared with normal human glial cells, suggesting that mTORC2 could be a better target that might diminish the expression of Hh-pathway proteins and reduce the CSCs without affecting normal astrocytes. Truly, we found that mTORC2 inhibitors (mahanine/Ku-0063794) were more effective toward CSCs and showed reduced levels of Gli1/Gli2 proteins with minimal toxicity to normal stem-like cells.

In summary, we have identified previously uncharacterized interactions between mTORC2 and the Hh pathway. Here we provide evidence that mTORC2 modulates cell division, angiogenesis, migration, invasion and stemness characteristics by activating the Hh pathway. Therefore, a potent mTORC2 inhibitor would be a better therapeutic, which can also reduce the CSCs. Furthermore, as mTOR lies downstream of several oncogenic and tumor-suppressor pathways and is a critical player in the tumor-microenvironment network, it would be possible to block several pathways by targeting mTORC2, which will be an additional advantage.

## Materials and methods

### Reagents

Iscove's modified Dulbecco's medium, fetal bovine serum (FBS) were from (Gibco, Life Technologies, Carlsbad, CA, USA), Lipofectamine LTX, plus reagent, matrigel, DMEM/F12, B27 supplement and N_2_ supplement were from Invitrogen (Carlsbad, CA, USA). Antibodies for mTOR(2983), phospho-mTOR (Ser2481) (2974), Rictor(9476), GSK-3*β*(9315), *β*-Actin(4970), Gli1(3538S), Ptch1(2468S), Sufu(2522S), Shh(2207S), Snail(3879S), Slug(9585S), VEGF(2463S), Cyclin D1(2978S), Cyclin D2(3741S), Cyclin E(81045S), Oct4(2840), Sox2(3579), Nanog(4903), Integrin *α*6(3750), HDAC3(2632S), rabbit IgG(3900S), HRP-conjugated anti-rabbit antibodies (7047S) and anti-mouse secondary antibodies (7076) were from Cell Signaling Technology (Danvers, MA, USA). Gli2(sc-28674), Gli3(sc-20688), Smo(sc-13943) antibodies, GANT-61, siRNAs against Gli2(sc-37913) and GSK-3*β*(sc-35527) were from Santa Cruz Biotechnology (Santa Cruz, CA, USA).

### Cell lines and culture condition

U87MG and LN229 human GBM cell lines were from ATCC (Manassas, VA, USA), cultured as described earlier.^13^ For specific experiments, cells (1 × 10^4^−1 × 10^6^) were treated with various inhibitors/mahanine/drugs under identical conditions. Mahanine was purified as described.^13^

U87MG cells (1 × 10^5^) were seeded on 6-cm low-attachment Petri dishes containing 3 ml of serum-free neural stem cell medium DMEM/F12, 20 ng/ml bFGF, 20 ng/ml EGF, 10 ng/ml heparin, B27 supplement and N_2_ supplement for sphere culture. Cells were incubated at 37 °C under 95% air, 5% CO_2_, 100% humidity and characterized by CD133 positivity, Oct4, Sox2, Nanog, Nestin expression and their colony formation ability. In parallel, human glial SVG cells were cultured similarly and used as normal glial stem cells.

### Plasmid knockdown/overexpression

Rictor_1 shRNA (Addgene plasmid#1853) and Rictor_2 shRNA (Addgene plasmid#1854) were a gift from David Sabatini.^30^ U87MG and LN229 cells were cultured in complete medium overnight. Individual target-specific siRNAs/shRNAs (2 *μ*g/ml) were transfected using lipofectamine Ltx and Plus reagents. These cells were used for following experiments in the presence or absence of different inhibitors after 24–36 h.

pCS2-MT GLI2 FL was a gift from Erich Roessler (Addgene plasmid#17648).^31^ For Rictor overexpression, we used vector encoding myc-tag wild-type Rictor (pRK-5/Rictor). Plasmid constructs were amplified and isolated using Qiaprep Spin Miniprep Kit (Qiagen). DNA (0.5–1 mg) was transfected using lipofectamine 2000.

### Immunoblotting

Untreated/treated cells with inhibitors/siRNA/shRNA/plasmids were harvested and lysed with sonication (Qsonica-LLC, XL-2000 series) keeping in ice-cold phosphate buffered saline and processed for western blotting.^32, 33^ Developed bands were either detected by X-ray plate or captured by Biorad ChemiDoc MP System (Bio-Rad, Hercules, CA, USA). Images were captured using Image Lab software (Biorad) version 5.2.1.

For the detection of mTORC2 formation and to identify the interactions between Rictor and Sufu, Rictor and Smo, and Sufu and Gli2, cells were cultured and coimmunoprecipitation was performed.^13^

### Real-time reverse transcription PCR analysis

Cells were cultured in different conditions and RNA was isolated using the RNeasy kit and quantified using a Nano Drop spectrophotometer. Complementary DNA was synthesized using the ImProm-II RT system (Promega, Madison, WI, USA); real-time PCR was performed using a DyNAmo Flash SYBR Green qPCR Kit. Relative amounts of target mRNAs were quantified using the LightCycler 96 (Roche) software with 18S rRNA as an internal control. The sequence of Primer is given in Table 1.

### Cell cycle analysis

Rictor was either overexpressed or silenced in LN229/U87MG cells and cultured for an additional 36 h and processed using the Cell Cycle Test Plus kit.^34^

### Cell viability assay

Stem-likes cells were treated with different inhibitors for 48 h, and cell viability was determined by MTT assay and PI positivity.^35^

### Gli reporter assay

Gli activity or regulation of Gli transcription was measured using a firefly luciferase-based Gli-reporter assay (8GLI-luciferase, Cignal reporter Gli). U87MG cells were transfected with negative and positive controls, Gli reporter and Gli reporter with Rictor shRNA. Similarly, LN229 cells were transfected with negative/positive controls, Gli reporter and Gli reporter with pRK-5 Rictor/Hh inhibitor. Cells were processed for dual luciferase assay after 48 h using the Promega Dual Luciferase Kit.

### Invasion/connective tube formation/migration assay

These assays were done with transfected/untransfected U87MG and LN229 cells as described earlier.^36, 37^

### Statistical analysis

All the data were from at least three independent experiments, and statistical analysis was performed using Graph Pad Prism 5. The differences between the groups were analyzed by two-tailed Student’s *t*-test or Mann–Whitney *U*-test. Standard error bars represent the standard deviation of the mean (±S.D.) and *P<0.05, **P<0.01, ***P<0.001 denoted the significant differences between the means of the untreated and treated cells or two test groups.

## Figures and Tables

**Figure 1:** Status of hedgehog pathway molecules in U87MG and LN229 cells. (**a**) Hypothesis: Is there any role of mTORC2 in regulating hedgehog pathway using GBM as a model system? (**b**) A representative immunoblot analysis (from three experiments) showing the status of the Gli1, Gli2^FL^, Gli3^Rep^, Ptch1, Sufu, Shh and Smo protein in U87MG and LN229 cells. *β*-Actin served as a loading control. For development of bands, Super Signal West Pico imaging system (Thermo-scientific) was used. (**c**) Fold change in mRNA expression of Gli1, Gli2, Gli3 and Ptch1 by real-time PCR analysis in LN229 cells relative to that of U87MG. Values are normalized against 18S rRNA expression (*n*=3 experiments). The data are presented as means ± SD of three independent experiments. Statistical significance compared with the control is indicated by **P<0.01 and ***P<0.001

**Figure 2:** mTORC2 regulates the expression of Gli1 and Gli2. U87MG cells were transfected with shRictor_1 and shRictor_2 shRNA (**a**–**c**) and LN229 cells were transfected with myc-tag wild-type Rictor (pRK-5/Rictor) for Rictor overexpression (**d**–**f**). After 36 h, cells were processed for western blotting, coimmunoprecipitation and real-time PCR analysis. RNA isolation kits were from Qiagen. (**a**) Representative immunoblot and coimmunoprecipitation of mTOR and Rictor confirmed reduced mTORC2 formation, as well as lower mTORC2 activity, as shown by decreased phosphorylation of mTOR at Ser2481 in U87MG cells after Rictor knockdown. (**b**) Real-time PCR analysis of Gli1, Gli2, Gli3 and Ptch1 mRNA expression in U87MG cells after mTORC2 disruption by shRictor_1 and shRictor_2 relative to that of untransfected cells. Values are normalized against 18S rRNA expression (*n*=3 experiments). (**c**) Representative immunoblot showing reduced Gli1, Gli2^FL^ and Ptch1 protein levels and increased Gli3^Rep^ upon Rictor knockdown in U87MG cells. However, there was no apparent change in protein level of Sufu, Smo and Shh. (**d**) Representative immunoblots and coimmunoprecipitation experiments confirmed enhanced mTORC2 formation, as well as increased mTORC2 activity, as shown by higher mTOR Ser2481 phosphorylation in Rictor-overexpressed LN229 cells. (**e**) Real-time PCR analysis of Gli1, Gli2, Gli3 and Ptch1 mRNA expression in LN229 cells after mTORC2 activation relative to that of untransfected cells. Values are normalized against 18S rRNA expression (*n*=3 experiments). (**f**) Representative immunoblots showing increased Gli1, Gli2^FL^, Ptch1 and decreased Gli3^Rep^ protein levels upon enhanced mTORC2 activity in LN229 cells, whereas Sufu, Shh and Smo protein levels remain almost equivalent. (**g**) Dual luciferase assay was performed using Gli reporter construct (Qiagen) in U87MG and LN229 cells. According to the manufacturer’s protocol, U87MG cells were transfected with negative control, positive control, Gli reporter and Gli reporter with Rictor shRNA. Similarly, LN229 cells were transfected with negative control, positive control, Gli reporter and Gli reporter with pRK-5Rictor/Hh inhibitor (GANT61, 100 nM). Cells were processed for dual luciferase assay after 48 h using the Promega Dual Luciferase Kit according to the manufacturer’s instructions. Graphs show the mean±S.D. percentage of a relative luciferase unit after normalizing by comparing with control (incubated with vehicle only). Experiments were done in triplicate. Statistical significance compared with the control is indicated by *P<0.05, **P<0.01 and ***P<0.001

**Figure 3:** mTORC2 regulates angiogenesis, invasion, migration and proliferation of cancer cells via the hedgehog pathway. U87MG cells were treated with either shRictor_1 and shRictor_2 or GANT61 (Gli2 inhibitor) (100 nM) for 24 h. Rictor was overexpressed in LN229 cells and treated similarly with GANT61 to perform the following experiments (A–L). (**a**) Real-time PCR analysis of Slug, Snail and VEGF mRNA expression in U87MG cells after mTORC2 disruption relative to that of shRictor-untransfected cells. Values are normalized against 18S rRNA expression (*n*=3 experiments). (**b**) Real-time PCR analysis of Slug, Snail and VEGF mRNA expression in LN229 cells after mTORC2 activation relative to that of untransfected cells. Values are normalized against 18S rRNA expression (*n*=3 experiments). (**c**) Representative immunoblots showing decreased Slug, Snail and VEGF protein levels upon reduced mTORC2 activity in U87MG cells, whereas all these protein levels were enhanced when mTORC2 activity was increased in LN229 cells. (**d**) Inverted light microscopic images showing reduced connective tubes formation between cellular colonies in Rictor-knocked-down and GANT61-treated U87MG cells compared with vehicle. Rictor-overexpressed LN229 cells exhibited increased connective tubes formation compared with untransfected cells, which was reduced in the presence of hedgehog inhibitor. (**e** and **f**) Treated or untreated U87MG or LN229 cells (5 × 10^4^) were suspended in medium without FBS (100 *μ*l) and added to the upper chamber of an insert (6.5 mm diameter, 8 *μ*m pore size; Becton Dickson). The insert was placed in a 24-well plate containing medium (700 *μ*l) with or without 10% FBS. Inverted light microscopic images of U87MG cells showing lower invasiveness when Rictor was knocked down or Gli2 activity was inhibited by GANT61. In contrast, LN229 cells showed increased invasion when Rictor was overexpressed. However, Rictor-overexpressed cells showed lower invasion in the presence of Gli2 inhibitor (**e**). Three randomly selected fields on the lower side of the insert were counted and graphically represented (*n*=3) (**f**). (**g** and **h**) U87MG and LN229 cells were cultured to >80% confluency in a six-well plate and treated with either shRictor or GANT61 for 24 h. Rictor-overexpressed LN229 cells were treated with GANT61. In every treated or untreated well, scratch was made by 2.5 *μ*l tips. Representative images showing the filling of gaps in each well after 36 h (**g**). Area of closure was calculated and graphically represented (*n*=3) (**h**). **(i** and **j**) Real-time PCR analysis of Rictor, cyclin D1, cyclin D2 and cyclin E mRNA expression in Rictor-knocked-down U87MG (**i**) and Rictor overexpressed LN229 cells (**j**) relative to that of untransfected cells. Values are normalized against 18S rRNA expression (*n*=3 experiments). (**k**) Representative immunoblots showed decreased proteins level of cyclin D1, cyclin D2 and cyclin E upon reduced mTORC2 activity in U87MG cells, whereas all these protein levels were enhanced upon increased mTORC2 activity in LN229 cells. (**l**) Flow cytometric analysis exhibited cell cycle arrest in Rictor-knocked-down U87MG cells and enhanced proliferation in Rictor-overexpressed LN229. y axis of the graphs is denoting the cell counts and x axis is denoting the DNA area. Cycle Test Plus kit (BD Bioscience) was used for cell cycle analysis. At least 20 000 cells were acquired in FACS and analyzed by CellQuest Pro software (BD FACSCalibur). The data are presented as means± SD of three independent experiments. Statistical significance compared with the control is indicated by *P<0.05, **P<0.01 and ***P<0.001

**Figure 4:** mTORC2 regulates the hedgehog pathway via GSK3*β*-dependent mechanism. (**a**) Rictor was either silenced in U87MG cells or overexpressed in LN229 cells. Representative immunoblots demonstrated increased or decreased GSK3*β* Ser9 phosphorylation upon Rictor-knocked-down or overexpression conditions. (**b**) Either Rictor alone or both Rictor and GSK3*β* were knocked down in U87MG cells. In parallel, GSK3*β* were also knocked down in LN229 cells before and after Rictor overexpression. Representative immunoblots showed enhanced Gli1, Gli2^FL^ and Ptch1 protein levels in Rictor-knocked-down U87MG cells. However, the levels of all three proteins were reduced when both Rictor and GSK3*β* were knocked down. In contrast, GSK3*β*-knocked-down LN229 exhibited increased level of all these proteins, whereas Rictor overexpression in GSK3*β*-knocked-down LN229 cells showed more enhanced protein levels. (**c**) LN229 cells were treated either with MG132 (inhibitor of ubiquitination) or GSK3*β* inhibitor SB17237 (Calbiochem USA) separately for 24 h. Representative immunoblot showed restoration of Gli2^FL^ protein in LN229 cells in a dose-dependent manner. (**d**) Gli2 was overexpressed in LN229 cells using vector encoding full-length Gli2. Real-time PCR analysis exhibited enhanced Gli1, Gli2, Ptch1, cyclin D1, cyclin D2, slug, snail and VEGF mRNA expression in Gli2-overexpressed LN229 cells relative to that of untransfected cells. Values are normalized against 18S rRNA expression (*n*=3 experiments). (**e**) Representative immunoblots showed enhancement of hedgehog pathway proteins and its downstream molecules upon Gli2 overexpression in LN229 cells. (**f**) Representative western blot showed lower nuclear accumulation of Gli1, Gli2^FL^ in LN229 cells compared with U87MG cells. HDAC3 and *β*-actin served as a loading control. (**g**) Representative western blot showed higher association of Gli2^FL^ and Sufu revealed by coimmunoprecipitation in LN229 cells. (**h**) Coimmunoprecipitation illustrated higher association of Smo with Rictor in U87MG cells and Rictor with Sufu in LN229. Statistical significance compared with the control is indicated by **P<0.01 and ***P<0.001

**Figure 5:** mTORC2 regulates stemness of GBM stem-like cells. (**a**) Representative immunoblot and coimmunoprecipitation demonstrated higher mTORC2 activity and formation as evidenced by increased mTOR Ser2481 phosphorylation and association with Rictor in CD133-positive stem-like cells derived from U87MG. APC-conjugated CD133 antibody was from Mylteni Biotech. (**b**) Immunoblot analysis showing enhanced mTOR Ser2481 and Gli2^FL^ in GBM stem-like cells compared with normal human glial stem cells. (**c**) Rictor was overexpressed in LN229 cells. Simultaneously, Gli2 was knocked down in Rictor-overexpressed LN229 cells and cultured in stem cell medium. Rictor-overexpressed cells showed enhanced neurosphere formation but were unable to form large colonies when Gli2 was knocked down. (**d**) Both the number of CD133-positive cells and their expression were higher in Rictor-overexpressed LN229 cells as revealed by flow cytometric analysis. (**e**) Representative western blots showed increased levels of Oct4, Sox2, Nanog, Integrin *α*6 and Nestin in Rictor-overexpressed LN229 cells. Nestin antibody was from Biolegend. Statistical significance compared with the control is indicated by *P<0.05

**Figure 6:** mTORC2 is a better therapeutic target for cancer stem-like cells. (**a**) Stem-like cells were treated separately with mTORC2 inhibitors (mahanine and Ku-0063794) (Sigma-Aldrich), GANT61 (Gli2 inhibitor), cyclopamine (Shh inhibitor) (Sigma-Aldrich) and temozolomide (DNA intercalator) (Sigma-Aldrich) at different doses. Cell viability was checked using Cell Proliferation Reagent WST-1 (Sigma-Aldrich). Only mahanine and KU exhibited significantly decreased viability of cancer stem-like cells in a dose-dependent manner. (**b**) U87MG cells were treated with different doses of mahanine for 24 h and processed for western blot analysis. The result showed that mahanine inhibited Gli1 and Gli2 proteins. (**c**) Mahanine-treated GBM stem-like cells exhibited reduced neurosphere formation in a dose-dependent manner. (**d**) Mahanine-treated stem-like cells showed significantly reduced number of CD133-positive cells and its expression, as revealed by flow cytometric analysis. (**e**) Stem-like cells demonstrated enhanced sensitivity toward mahanine in a dose-dependent manner, as determined by PI positivity analysis using flow cytometry. (**f**) Mahanine showed minimal toxicity to normal glial cells compared with cancer stem-like cells. (**g**) Pictorial representation of summary of the events describing cross talk between mTORC2, Hh pathway and stemness characteristics in GBM. Statistical significance compared with the control is indicated by **P<0.01 and ***P<0.001

**Table 1:** Primer details

**Primers**	**Sequence**
RICTOR F	GGAAGCCTGTTGATGGTGAT
RICTOR R	GGCAGCCTGTTTTATGGTGT
GLI1 F	GTGCAAGTCAAGCCAGAACA
GLI1 R	ATAGGGGCCTGACTGGAGAT
GLI2 F	TTTATGGGCATCCTCTCTGG
GLI2 R	AAGGCTGGAAAGCACTGTGT
GLI3 F	TCCCAGCGCTTTCTACATCT
GLI3 R	CTTTGTCGTGGACCCATTCT
PTCH1 F	TCCCAGCGCTTTCTACATCT
PTCH1 R	CTTTGTCGTGGACCCATTCT
CYCLIN D1 F	CCTAAGTTCGGTTCCGATGA
CYCLIN D1 R	ACGTCAGCCTCCACACTCTT
CYCLIN D2 F	ATTGGCATGTCTGGTTCACA
CYCLIN D2 R	GCCAGATACCAGAAGCGAAG
CYCLIN E F	AGCGGTAAGAAGCAGAGCAG
CYCLIN E R	TTTGATGCCATCCACAGAAA
VEGFA F	AGGCCAGCACATAGGAGAGA
VEGFA R	TTTCTTGCGCTTTCGTTTTT
SNAIL F	GAGGACAGTGGGAAAGGCTC
SNAIL R	TGGCTTCGGATGTGCATCTT
SLUG F	CATCTTTGGGGCGAGTGAGT
SLUG R	GGCCAGCCCAGAAAAAGTTG
